# Cytokine Levels and Severity of Illness Scoring Systems to Predict Mortality in COVID-19 Infection

**DOI:** 10.3390/healthcare11030387

**Published:** 2023-01-29

**Authors:** Sevda Onuk, Hilal Sipahioğlu, Samet Karahan, Ali Yeşiltepe, Sibel Kuzugüden, Aycan Karabulut, Zehra Beştepe Dursun, Aynur Akın

**Affiliations:** 1 Department of Intensive Care, Kayseri City Education and Research Hospital, 38080 Kayseri, Turkey; 2 Department of Internal Medicine, Division of Rheumatology, Kayseri City Education and Research Hospital, 38080 Kayseri, Turkey; 3 Department of Clinical Biochemistry, Kayseri City Education and Research Hospital, 38080 Kayseri, Turkey; 4 Department of Internal Medicine, Kayseri City Education and Research Hospital, 38080 Kayseri, Turkey; 5 Department of Infectious Disease, Kayseri City Education and Research Hospital, 38080 Kayseri, Turkey; 6 Department of Medicine, Division of Anesthesiology and Reanimation Intensive Care, Erciyes University, 38039 Kayseri, Turkey

**Keywords:** COVID-19, SARS-CoV-2, cytokines, comorbidity, APACHE II, Sequential Organ Failure Assessment Score

## Abstract

Various scoring systems and cytokines have been cited as predicting disease severity in COVID-19 infection. This study analyzed the link between mortality rate, levels of cytokines, and scoring systems such as the Glasgow Coma Scale (GCS), Acute Physiologic Assessment and Chronic Health Evaluation II (APACHE II), Sequential Organ Failure Assessment (SOFA), and Charlson Comorbidity Index in patients infected with COVID-19. Adult patients infected with COVID-19 were followed up in the intensive care unit (ICU) and analyzed prospectively. We measured serum cytokine levels (Interleukin-10 (IL-10), Interleukin-8 (IL-8), Interleukin-6 (IL-6), Interleukin-1β (IL-1β), tumor necrosis factor-alpha (TNF-α) and High mobility group box 1 (HMGB-1)) and recorded GCS, APACHE II, SOFA, and Charlson comorbidity index scores on admission to the ICU. Receiver operating curve (ROC) analysis was performed to predict mortality from IL-1β, IL-6 IL-10, IL-8, TNF-α, and HMGB-1 values. Study participants were grouped as follows: Group A, survivors, and Group B, deceased, during the 28-day follow-up. The mean age was 65.69 (±13.56) in Group A (*n* = 36) and 70.85 (±10.06) in Group B (*n* = 27). The female/male ratio was 23/40. Age, sex, body mass index (BMI), comorbid illnesses, GCS, APACHE II, SOFA, and Charlson scores, duration of hospitalization or ICU admission, therapeutic choices, and lymphocyte, PMNL, NLR, platelet, D-dimer, fibrinogen, GGT, CRP, procalcitonin, and lactate levels were similar between the groups. The frequency of acute kidney injury (AKI) was higher in Group B (*p* = 0.005). Serum IL-10, IL-8, IL-6, IL-1β, TNF-α, HMGB-1, ferritin, and LDH values were higher, and PaO_2_/FiO_2_ was lower in Group B than in Group A. ROC analysis showed that there was an association between serum IL-1β (>1015.7), serum IL-6 (>116.7), serum IL-8 (>258.4), serum IL-10 (>247.5), serum TNF-α (>280.7), and serum HMGB-1 (>23.5) and mortality. AKI gave rise to a greater risk of mortality (odds ratio: 7.081, *p* = 0.014). Mortality was associated with serum IL-10, IL-8, IL-6, IL-1β, TNF-α, and HMGB-1 but not with GCS, APACHE II, SOFA, or Charlson comorbidity index scores. AKI increased the risk of mortality by seven times. Our findings suggest that cytokine levels (serum IL-10, IL-8, IL-6, IL-1β, TNF-α, and HMGB-1) were predictors of mortality in COVID-19 infection. In addition, our results might give an opinion about the course of COVID-19 infection.

## 1. Introduction

COVID-19 infection has affected people worldwide. On the 11th of March 2020, COVID-19 was designated a pandemic by the World Health Organization (WHO); to date, it has affected approximately 6.5 million people worldwide [1]. Research data have shown that the resultant mortality rate of SARS-CoV-2 infection is high in the general population [1,2]. The Turkish Ministry of Health has declared that more than 16 million have been impacted by SARS-CoV-2 infection, and of these, some 101,000 plus individuals in Türkiye have died as of October 2022 [3]. However, there was no appropriate therapy protocol for COVID-19 infection. In the intensive care unit, patients with COVID-19 infection usually had hypoxia or radiographic evidence of pneumonia and were treated with high-flow oxygen/invasive or non-invasive ventilation. When patients experienced worsening respiratory functions, the assessment of interleukin-6 (IL-6), D-dimer, ferritin, fibrinogen, C-reactive protein, and lactate dehydrogenase values was suggested [4].

Cytokine storm and macrophage activation were shown to be important factors with respect to SARS-CoV-2 infection pathogenesis [5]. Cytokine storms resulting from COVID-19 infection may affect multiple organs, give rise to acute respiratory distress, or disseminate intravascular coagulation [6]. Increases in various cytokine concentrations such as IL-10, IL-8, Il-6, IL-1β, and TNF-α were observationally linked with infection severity and/or mortality [6,7,8,9,10,11]. Therapeutic interventions have been developed against these cytokines [6,7,8].

The Charlson comorbidity index (CCI) was developed as a prognostic index that predicts mortality based on several comorbidities in surgical patients [12,13]. It has been studied in patients with various cancers as well as in COVID-19 infection [14,15,16,17,18,19]. CCI in COVID-19 infection was found to be a predictor of not just mortality but also respiratory failure and admission to the ICU [18,19,20,21]. Additional predictors of mortality in patients infected with COVID-19 included the Sequential Organ Failure Assessment (SOFA) and the Acute Physiology and Chronic Health Evaluation II (APACHE II) scoring system and other indexes [22,23,24,25,26,27].

We hypothesized that inflammatory cytokine levels and the severity of illness of scoring systems might predict the mortality in COVID-19 infection. This research sought to analyze the link between mortality, cytokine levels, and the Glasgow Coma Scale (GCS), Acute Physiologic Assessment and Chronic Health Evaluation II (APACHE II), Sequential Organ Failure Assessment (SOFA), and Charlson Comorbidity Index scoring systems.

## 2. Materials and Methods

### 2.1. Study Design

This study, which was prospective in nature, was conducted in Kayseri City Training and Education Hospital and received approval from the local Ethics Committee of Kayseri City Training and Education Hospital Ethic Committee (Number: 20.05.2021/396). This research was undertaken per the principles set out by the Helsinki Declaration (1964) and the following amendments. Informed consent was obtained from all individual participants included in the study.

The adult patients diagnosed with COVID-19 infection and followed up in the ICU in Kayseri City Training and Education Hospital between May 2021 and March 2022 were analyzed prospectively. A COVID-19 diagnosis was carried out through PCR testing and analyzed from nasal swab samples taken from patients suspected of being infected with COVID-19. We also included patients whose thorax computed tomography was positive for COVID-19 infection but whose PCR test was negative (3). All patients underwent clinical and radiological evaluation. Those for whom data were missing; those who were younger (<18 years old), pregnant, or treated with immunosuppressive drugs before ICU admission; or had a history of chronic renal failure, congenital or acquired immunodeficiency were not included in the study.

### 2.2. Data Collection

Age, body mass index (BMI) and sex; clinical parameters (symptoms, comorbid illnesses (hypertension, type 2 diabetes mellitus, coronary artery disease, chronic pulmonary disease, cerebrovascular accident, and liver disease), duration of hospitalization (days), duration of ICU admission (days)); PaO_2_/FiO_2_ ratio; laboratory findings (ferritin, C-reactive protein (CRP), procalcitonin, fibrinogen, gamma-glutamyltransferase (GGT), D-dimer, lactate dehydrogenase (LDH) and lactate levels, lymphocyte, neutrophil (PMNL) and platelet counts, and the ratio of neutrophil to lymphocyte (NLR)); and therapeutic choices (tocilizumab, dexamethasone, methylprednisolone) were recorded using electronic and written patient files.

Complete blood count was studied with an automated analyzer.

Serum cytokines levels (IL-10, IL-8, Il-6, IL-1β, TNF-α, and high-mobility group box 1 (HMGB-1)) were measured only once upon ICU admission. Requisite blood samples were obtained and placed in a gel tube and preserved at −80 °C after centrifugation. Serum cytokine levels were measured at the biochemistry laboratory by the ELISA method as per the manufacturer’s instructions.

GCS, APACHE II, SOFA, and Charlson comorbidity index scores of the study sample were evaluated upon admission to the ICU [12,13,28,29].

### 2.3. Patient Groups

The patients were grouped based on mortality: Group A, survivors, consisted of patients who survived beyond the 28-day follow-up; and Group B, deceased, consisted of the patients who died during the 28-day follow-up. We compared demographic, clinical, and laboratory parameters between the groups.

### 2.4. Statistical Analysis

IBM SPSS Statistics Standard Concurrent User V 26 package program (IBM Corp., Armonk, New York, NY, USA) was employed for data analysis purposes. An evaluation of quantitative data conformity to normal distribution was conducted using the Shapiro–Wilk test, while the Levene test was utilized to evaluate variance homogeneity. When comparing quantitative data from two independent groups, we used a parametric t-test and a nonparametric Mann–Whitney U test. A comparison of categorical variables was conducted with the Pearson chi-square test. The correlation between cytokine levels and biochemical parameters was analyzed using Spearman’s correlation analysis. To detect the relationship between the real classification of the procedure’s success and the classification made by the cut-off values, sensitivity, and specificity ratios, positive and negative predictive values were expressed by ROC (receiver operating curve) analysis. An analysis of the factors affecting mortality was undertaken using multiple binary logistic regression and the backward stepwise (Wald) method. Median (minimum–maximum) and mean (standard deviation) values, as well as the interquartile range (IQR), were used in the description of quantitative data, with the number (*n*) and percentage (%) representing the categorical variables in the tables. *p* < 0.05 and a confidence level of 95% were considered indicators of statistical significance.

Post-power analysis was performed in G-Power 3.1 software. For inflammatory cytokines (serum IL-1β, IL-6, IL-8, IL10, TNF-α, HMGB-1) values, the range of post-power strength was calculated as 82.3–94.6% with a medium effect size (d = 0.5).

## 3. Results

The mean age was 65.69 (±13.56) in Group A (*n* = 36) and 70.85 ± 10.06 in Group B (*n* = 27) (*p* = 0.102). In total (*n* = 63), the female/male ratio was 23/40. Sex, BMI, and comorbidity illnesses were similar in Groups A and B. GCS, APACHE II, SOFA, and Charlson comorbidity index scores were similar in Groups A and B. The frequency of acute kidney injury (AKI) was higher in Group B (*p* = 0.005). Duration of hospitalization, duration of ICU admission, and therapeutic choices was similar in Groups A and B (Table 1).

Higher levels of serum IL-10, IL-8, Il-6, IL-1β, TNF-α, and HMGB-1 were observed in Group B compared to Group A. Ferritin, and LDH levels were higher, and PaO_2_/FiO_2_ levels were lower, in Group B than those in Group A. Lymphocyte, PMNL, NLR, platelet, D-dimer, fibrinogen, GGT, CRP, procalcitonin, and lactate levels were similar in Groups A and B (Table 2). Serum cytokine levels and blood count or biochemical parameters in Group B showed no correlation. Serum IL-6 concentrations had a positive correlation with fibrinogen (Rho: 0.525, *p* = 0.001), ferritin (Rho: 0.352, *p* = 0.035), and CRP (Rho: 0.452, *p* = 0.006) levels in Group A.

ROC analysis showed that there was an association between serum IL-1β (>1015.7), serum IL-6 (>116.7), serum IL-8 (>258.4), serum IL-10 (>247.5), serum TNF-α (>280.7), and serum HMGB-1 (>23.5) and mortality. Among the cytokines, serum IL-1β was the most sensitive, and serum TNF-α was the most specific cytokine predicting mortality. The AUC value of TNF-α was higher than that of the other cytokines (Table 3 and Figure 1).

Logistic regression analysis showed that AKI increased the risk of mortality (odds ratio: 7.081, *p* = 0.014) (Table 4).

## 4. Discussion

We found that serum IL-10, Il-8, IL-6, IL-1β, TNF-α, and HMGB-1 levels were higher in patients who had died but that GCS, APACHE II, SOFA, and Charlson comorbidity index scores were not associated with 28-day mortality. AKI increased the risk of mortality by about seven times.

White blood cells and other cell types secrete cytokines and provide activation of defense mechanisms. Various cell types can be acted on by the same cytokines or a single cytokine secreted from different cells [8]. One cytokine may stimulate target cells to secrete additional cytokines, and they fight together against infection. In addition, pleiotropic effects, cascade induction, and synergistic effects of elevated levels of cytokines may harm the tissues [8]. In COVID-19, cytokine storm actions, which may result from the release of TNF-α, interferon, and interleukins, may give rise to multi-organ damage, acute respiratory distress syndrome, pulmonary complications, or disseminated intravascular coagulation infection [6,7,8].

Elevated levels of inflammatory mediators were seen to be associated with a worse prognosis for COVID-19 infection [6,7,8]. In one study of 52 individuals infected with COVID-19, the maximum concentrations of plasma cytokines (IL-2, IL-5, IL-17, IL-8, IL-10, IL-6, IL-12p70, and IFN-γ) were found to be significantly higher in those who had died than in those who had survived [30]. IL-6, IL-8, and IL-5 values measured previously were also seen to be higher in those who had died. In that study, cytokine levels were shown to be associated with disease duration [30]. We proposed that the need for ICU admission might indicate disease progression and, therefore, be associated with elevated cytokine levels. Therefore, we measured cytokine levels only upon admission of the patients to the ICU, not during follow-up. We assessed mortality according to the number of deceased patients in the 28-day period of ICU admission. Another study also showed that COVID-19 severity was linked with higher levels of proinflammatory cytokines in the first waves of the pandemic, with IL-8, IL-6, and IL-10 having the highest AUC values [31]. In addition, Jafrin et al. [32] performed a meta-analysis and systematic review of 147 clinical studies investigating IL-6 and IL-10 in 31,909 patients with COVID-19 infection. It was reported that IL-6 concentrations were significantly higher in deceased patients compared to survived patients (mean difference: 42.11; *p* < 0.001; 95% CI: 36.86, 47.36). In contrast, IL-10 values were significantly higher in the dead study participants than in the survived participants (mean difference: 4.79; *p* < 0.001; 95% CI: 2.83, 6.75). In addition, the authors suggested that the measurement of IL-6 and IL-10 concentrations should be an option to predict mortality in COVID-19.

We did not include a control group and found patient cytokine levels were elevated in the presence of COVID-19. We measured proinflammatory cytokines serum TNF-α, IL-6, IL-1β, IL-8, and anti-inflammatory cytokine IL-10. COVID-19 infection may trigger a severe immune-inflammatory response. Infection progression is affected by the balance in levels between proinflammatory and anti-inflammatory cytokines; however, with respect to anti-inflammatory cytokines, their role still remains unclear. In some previous reports, both proinflammatory and anti-inflammatory cytokines (IL-13 and IL-10) were shown to be increased and predictive of disease severity [30,31,32,33,34,35]. Contrast findings regarding the association of anti-inflammatory cytokine levels (IL-10, IL-4, IL-13) with the severity of COVID-19 infection were also reported [36,37]. Increased IL-10 levels may be a feedback modulator response to elevated IFN-γ and IL-6 levels, may not play a protective role, and suggest a latent effect acting on the cytokine storm [33,38]. IL-13 was observed to disrupt type 2 pneumocyte stem cell activity, and IL-4 level was found to be increased in patients followed up in the ICU [33]. Where both anti-inflammatory and proinflammatory cytokine levels are elevated, the cumulative effect may affect the cytokine storm’s course. The effect of anti-inflammatory cytokines should be explained in future studies. Milen kovic et al. performed a retrospective cohort study in 318 COVID-19 patients treated in ICU to predict hospital mortality with D-dimer, CRP, PCT, and IL-6 values. Similarly, it was found that non-survivor patients had significantly elevated IL-6, D-Dimer, CRP, and PCT values than non-survivor patients. In addition, IL-6 was a statistically significant predictor of hospital mortality, and the cut-off value of IL-6 was found to be 74.98 pg/mL (sensitivity 69.7%, specify 62.7%) [39]. Ozger et al. [40] performed a prospective study in 37 COVID-19 patients predicting mortality with serial IL-6, IL-7, IL-10, IL-15, IL-27 IP-10, MCP-1, and GCSF values. Similar to our study, non-survivor patients with COVID-19 infection had significantly higher IL-6 and IL-10 concentrations compared to survivor patients with COVID-19 on hospital admission. In addition, the cut-off value of IL-6 concentrations was 48.8 (AUC: 0.85, 95% Cl: 0.65 to 0.92) and 53.7 (AUC: 0.92, 95% Cl: 0.78–0.98) pg/mL on hospital admission and 3rd day of hospitalization. Furthermore, the cut-off value of IL-10 values were 24.4 (AUC: 0.88, 95% Cl: 0.73–0.96) and 15.0 (AUC: 0.93, 95% Cl: 0.80–0.99) pg/mL on hospital admission and 3rd day after hospital admission.

HMGB-1 protein is localized in the nucleus of most cells, may be secreted into the extracellular medium, and contributes to inflammation as well as to the pathogenesis of different inflammatory and autoimmune diseases [41]. The cytolytic effect of COVID-19 infection may lead to the release of HMGB-1 due to nuclear damage [42]. Elevated serum HMGB-1 levels in infected patients, both by activating the release of inflammatory cytokines and mediating RAGE, TLR, or MAPK signaling, may be associated with severe disease, cytokine storm, acute lung injury, and mortality [42,43,44]. We showed that HMGB-1 was associated with mortality with relatively lower specificity, and it was not included in the multivariate analysis indicating predictors of mortality.

Increased levels of biochemical parameters, such as procalcitonin, fibrinogen, CRP, or hemogram parameters, were linked with infection severity, ICU admission as well as mortality in previous studies [45,46,47,48]. In contrast, our findings suggested that neither fibrinogen, procalcitonin levels nor blood count parameters such as lymphocyte, PMNL, and NLR were associated with mortality. We found that IL-6 was positively correlated with biochemical markers only in patients who survived beyond 28 days, but no correlation was found in deceased patients.

Studies investigating cytokine levels together with the Charlson, APACHE II, or SOFA scores are limited. In one study, IL-1β and HGF (hepatocyte growth factor) were reported to be positively correlated with the severity of the disease defined by the APACHE II score during the first week of COVID-19 infection; however, there was a negative correlation between chemokine (C-X-C motif) ligand (CXCL) 1 (GRO-alfa), IL-9, TNF-α and TNF-β and disease severity [33]. With respect to cytokine levels and GCS, APACHE II, SOFA, or Charlson scores, no correlation analysis was undertaken.

The Charlson comorbidity index (CCI) has been validated for use in the prediction of mortality based on comorbidities [12,13,14]. In one study, a prediction model consisting of age-adjusted CCI, CRB score, and basal oxygen saturation was shown to be predictive of mortality in those infected with COVID-19 [18]. Similar findings were also reported in other studies [19,20,21]. An analysis of older patients infected with COVID-19 found that Elixhauser Comorbidity Index and quick SOFA scores were helpful in determining high-risk patients; however, CCI was not a predictor for mortality in multivariate analysis [20]. In another study, the CCI score was shown to be weakly correlated with the chance of mortality or ventilation support [47,49]. In some studies, the mortality risk was higher, where CCI scores were elevated in those infected with COVID-19 [50,51]. With regard to the APACHE II score, Ayvat et al. found it to be predictive of mortality in those infected with COVID-19 and followed up in the ICU, but that SOFA or GCS scores did not predict mortality [22]. Conflicting results were reported regarding the superiority of SOFA and APACHE II scores compared to each other [22,52,53]. Our findings suggest that these scores were not associated with mortality. This might result from the inclusion of patients in critical care settings or the relatively low number of patients. We analyzed survival on the 28th day of follow-up; however, in-hospital or in-ICU mortality, or longer duration (60th day) of follow-up, were analyzed in previous studies [23,24,54]. This might also contribute to the lack of association between the scoring systems and mortality in our study. We evaluated these scores upon admission to the ICU; however, the APACHE II score was periodically evaluated in one study analyzing COVID-19 infection [48,55].

Regarding acute kidney injury and elevated serum creatinine levels, an association with the severity of COVID-19 infection has been shown [35]. We found that AKI increased the risk of mortality by about seven times. TNF-α and IL-1β levels were also input into the model, indicating the predictors of mortality, but these were not clinically significant predictors for mortality in our study. This might be due to our sample size. We could not measure the levels of cytokines during follow-up in the ICU. The time of elevation of cytokine level and the persistence of elevation may depend on the type of cytokine. In some studies, IL-6, IL-8, and IL-10 levels were shown to rise in non-survivor patients with COVID-19 infection persistently; however, IL-2 and IL-4 levels were higher in the recovery period [37,56]. Therefore, measurement of a broad range of cytokines during follow-up would be beneficial. In one study, combining the effect of IL-8, IL-6, and IL-10 was shown to predict the severity of COVID-19 infection [57].

On the other hand, a brief report by Capalbo et al. [4] suggested that dexamethasone or tocilizumab should be beneficial for hospitalized patients with COVID-19 in ICU. Some study participants in our study were treated with dexamethasone or tocilizumab. Those participants had similar serum IL-1β, IL-6, IL-8, IL10, TNF-α, and HMGB-1 concentrations compared to participants treated with dexamethasone or tocilizumab therapy. Zhang et al. [58]. Performed a meta-analysis of 222 randomized controlled studies with 102,950 patients diagnosed with COVID-19 investigating the effects of different COVID-19 treatments, such as tocilizumab, dexamethasone, imatinib, intravenous immunoglobulin, etc., on poor clinical outcomes (mortality, mechanical ventilation, hospital discharge, and viral clearance). The authors found that patients treated with tocilizumab therapy had a significantly decreased mortality rate compared to patients who received tocilizumab treatment (OR 0.85, 95% CI: 0.77, 0.95) in 10 randomized controlled studies including 3401 patients with COVID-19. In addition, it was indicated that the effect of dexamethasone therapy on COVID-19 infection was conflicting.

## 5. Strength and Limitations

We analyzed a considerable number of both proinflammatory and anti-inflammatory cytokines in the prediction of mortality in COVID-19 infection. HMGB-1 levels were studied less in previous studies analyzing COVID-19 infection. We measured HMGB-1 levels and found higher levels in patients who had died. We evaluated the GCS, APACHE, SOFA, and Charlson scoring systems together with cytokine measurements. The principal limitation of the current study is the number of patients included. We measured cytokine levels and evaluated scoring systems only upon admission of the patients to the ICU, but we could not obtain repeated measurements or evaluations during the follow-up. We cannot generalize our results to all patients with COVID-19 infection in ICU. Future studies should be addressed with continuous measurements of cytokines in COVID-19 infection. In addition, studies with large samples investigating inflammatory cytokines levels in patients with COVID-19 are needed. The effect of different medical therapy should be examined in COVID-19 infection requiring ICU treatment.

## 6. Conclusions

We analyzed both proinflammatory and anti-inflammatory cytokine levels, in addition to scoring systems, in those infected with COVID-19 upon admission to the ICU. There was an association between serum IL-1β, Il-6, IL-8, IL-10, TNF-α, and HMGB-1 with mortality. We stated that AKI increased the risk of mortality by about seven times in patients with COVID-19 infection. To our knowledge, the number of studies analyzing HMGB-1 in COVID-19 infection is limited. GCS, APACHE II, SOFA, and Charlson scores were not associated with mortality. It would be beneficial to repeat the measurements of a broad range of cytokines as well as evaluations of scoring systems both at admission and during follow-up.

## Figures and Tables

**Figure 1:** ROC analysis curve demonstrating the association of cytokines with mortality.

**Table 1:** Comparison of demographic and clinical parameters among the groups.

	Groups		Test Statistics	
	Group A (Survived) *n* = 36	Group B (Died) *n* = 27	Test Value	*p* Value
Age $\bar{x}$ ± sd M (min–max)	65.69 ± 13.56 64.5 (45.0–43.0)	70.85 ± 10.06 73.0 (35.0–53.0)	*t* = 1.661	0.102
Sex *n* (%) Female Male	17 (73.9) 19 (47.5)	6 (26.1) 21 (52.5)	χ^2^ = 4.160	0.064
BMI $\bar{x}$ ± sd	26.94 ±4.50	28.12 ± 3.81	*t* = 1.097	0.277
Type 2 diabetes mellitus Absent Present	22 (59.5) 14 (53.8)	15 (40.5) 12 (46.2)	χ^2^ = 0.196	0.797
Hypertension Absent Present	18 (62.1) 18 (52.9)	11 (37.9) 16 (47.1)	χ^2^ = 0.532	0.610
Coronary artery disease Absent Present	26 (55.3) 10 (62.5)	21 (44.7) 6 (37.5)	χ^2^ = 0.251	0.772
Cerebrovascular accident Absent Present	32 (56.1) 4 (66.7)	25 (43.9) 2 (33.3)	χ^2^ = 0.246	0.693
Chronic pulmonary disease Absent Present	29 (58.0) 7 (53.8)	21 (42.0) 6 (46.2)	χ^2^ = 0.073	>0.999
Liver disease Absent Present	36 (58.1) 0 (0.0)	26 (41.9) 1 (100.0)	χ^2^ = 1.355	0.429
APACHE II score M (IQR)	10.0 (4.75)	11.0 (9.0)	z = 1.689	0.091
SOFA score M (IQR)	4.0 (1.0)	5.0 (3.0)	z = 1.217	0.224
GCS score M (IQR)	15.0 (2.0)	15.0 (1.0)	z = 1.064	0.287
Charlson comorbidity index score M (IQR)	4.0 (2.75)	4.0 (4.0)	z = 1.073	0.283
AKI Absent Present	31 (68.9) 5 (27.8)	14 (31.1) 13 (72.2)	χ^2^ = 8.873	0.005
Duration of hospitalization M (IQR)	19.5 (16.75)	15.0 (18.0)	z = 1.237	0.216
Duration of ICU admission M (IQR)	10.50 (8.0)	11.0 (12.0)	z = 1.351	0.177
Tocilizumab therapy Absent Present	31 (58.5) 5 (50.0)	22 (41.5) 5 (50.0)	χ^2^ = 0.248	0.733
Dexamethasone therapy M (IQR)	16.0 (8.0)	16.0 (8.0)	z = 0.612	0.594
Methylprednisolone therapy M (IQR)	40.0 (40.0)	60.0 (129)	z = 0.055	>0.999

%: row percent, $\bar{x}$: mean, sd: standard deviation, M: median, IQR: interquartile range, *t*: independent samples *t*-test, z: Mann–Whitney U test, χ^2^: chi-square test.

**Table 2:** Comparison of blood count, biochemical parameters, and cytokine levels among the groups.

	Groups		Test Statistics	
	Group A (Survived) *n* = 36 M (IQR)	Group B (Died) *n* = 27 M (IQR)	z Value	*p* Value
Lymphocyte	0.77 (1.13)	0.66 (0.52)	0.896	0.370
PMNL	9.74 (8.31)	8.79 (9.05)	0.451	0.652
NLR	10.67 (14.50)	15.50 (15.09)	1.278	0.201
Platelet	242.50 (114.0)	220.0 (105.0)	1.111	0.266
D-dimer	1650.0 (2844.50)	2230.0 (2716.0)	0.354	0.723
Fibrinogen	5830.0 (3495.0)	6650.0 (1560.0)	1.375	0.169
Ferritin	459.50 (790.25)	863.0 (1463.0)	2.833	0.005
LDH	370.50 (305.5)	553.0 (314.0)	2.834	0.005
GGT	29.0 (30.32)	39.0 (28.0)	1.362	0.173
CRP	117.0 (156.02)	96.0 (149.0)	0.361	0.718
Procalcitonin	0.18 (0.86)	0.55 (1.25)	1.459	0.145
Lactate	1.45 (1.25)	1.60 (1.0)	0.612	0.540
PaO_2_/FiO_2_	82.42 (139.50)	71.42 (27.78)	2.709	0.007
IL-1β	1093.50 (611.64)	1312.70 (1114.86)	2.236	0.025
IL-6	94.15 (37.08)	133.54 (120.94)	2.479	0.013
IL-8	198.39 (68.89)	263.68 (272.36)	2.660	0.008
IL-10	212.36 (133.75)	263.25 (364.76)	2.222	0.026
TNF-α	154.43 (69.52)	193.85 (182.10)	2.868	0.004
HMGB-1	20.99 (9.68)	26.0 (20.65)	2.201	0.028

M: median, IQR: interquartile range, z: Mann–Whitney U test.

**Table 3:** ROC analysis demonstrating cut-off values of cytokines associated with mortality.

	AUC (%95 CI)	*p* Value	Cut-Off	Sensitivity (%95 CI)	Specificity (%95 CI)
TNF-α	0.712 (0.585–0.820)	0.001	>280.7	37.0 (19.4–57.4)	100.0 (90.3–100.0)
IL-8	0.697 (0.568–0.807)	0.004	>258.4	51.8 (31.9–71.4)	80.5 (64.0–91.8)
IL-6	0.684 (0.554–0.795)	0.010	>116.7	55.5 (35.3–74.5)	83.3 (67.2–93.6)
IL-1β	0.666 (0.536–0.780)	0.018	>1015.7	88.8 (70.8–97.6)	41.6 (25.5–59.2)
IL-10	0.665 (0.534–0.779)	0.024	>247.5	55.5 (35.3–74.5)	80.5 (64.0–91.8)
HMGB-1	0.663 (0.533–0.777)	0.021	>23.5	59.2 (38.8–77.6)	69.4 (51.9–83.7)

AUC: area under the curve, CI: confidence interval.

**Table 4:** Logistic regression analysis demonstrating the factors predicting mortality.

	Regression Coefficients			
	*p*	Odds Ratio	95% CI	
			Lower	Upper
Constant	0.001	0.016		
AKI	0.014	7.081	1.482	33.834
IL-1β	0.016	1.005	1.001	1.009
TNF-α	0.004	1.047	1.015	1.080
Ferritin	0.016	1.001	1.000	1.002

Variables entered in step 1: Sex, AKI, APACHE II, IL-1β, IL-6, IL-8, IL-10, TNF-α, HMGB-1, ferritin, LDH. Elimination method: Backward Wald model summary: Hosmer and Lemeshov test χ^2^ = 7.028; *p* = 0.534; Nagelkerke *R*^2^ = 0.572, CI: confidence interval.

## Data Availability

The data that support the findings of this study are available from the corresponding author upon reasonable request.
